This article has been retracted.

# Clinical Analysis of 85 Cases of External Auditory Canal Cholesteatoma Surgery under Specialized Endoscopy

**DOI:** 10.1155/2022/9190241

**Published:** 2022-10-05

**Authors:** Yanan Guo, Minfei Qian, Jiping Li, Ji Xu, Hao Chen, Hua Zhang

**Affiliations:** Department of Otolaryngology, Ren Ji Hospital, Shanghai Jiao Tong University School of Medicine, Shanghai 200127, China

## Abstract

**Objective:**

To investigate the clinical characteristics, surgical experience, and surgical outcomes of external auditory canal cholesteatoma (EACC) surgery under endoscopic otolaryngoscopy.

**Methods:**

A retrospective analysis of 85 EACC cases admitted to the Department of Otolaryngology, Renji Hospital, Shanghai Jiaotong University School of Medicine, from January 2016 to February 2021 was performed, followed by retrospective analysis of clinical data to explore the feasibility and clinical characteristics of all-oral endoscopic EACC surgery. A total of 85 EACC patients (90 ears) with a mean age of 49.93 ± 14.87 years were included in the study. According to Udayabhanu staging, 43 ears (47.78%) were stage I, 40 ears (44.44%) were stage II, and 7 ears (7.78%) were stage III. All patients underwent transendoscopic surgery.

**Results:**

79 ears (87.78%) underwent endoscopic EACC resection alone (+external auditory canal tumor resection/tympanostomy tube insertion), 9 ears (10%) underwent endoscopic EACC resection+tympanostomy+tympanoplasty, 1 ear (1.11%) underwent endoscopic EACC resection+tympanoplasty, and 2 ears (2.22%) underwent EACC resection+otolaryngotomy+tympanoplasty+auditory chain reconstruction endoscopically. Of these, 7 ears (7.78%) underwent auricular cartilage-chondroplasty and 2 ears (2.22%) underwent auricular cartilage membrane repair. All patients were reviewed at 1 week, 2 weeks, 1 month, 3 months, 6 months, and 1 year postoperatively. One patient with stage II external auditory atresia had a recurrence after 6 months and underwent endoscopic ear surgery (ESS) again. One patient with stage 2 atresia recurred after 1 year and again underwent endoscopic ear surgery. The rest of the patients recovered well after the surgery, and the grafts healed well.

**Conclusion:**

EACC surgery through the external ear canal under a dedicated endoscope is a safe, reliable, and effective method. Patients with stage I and II external auditory canal cholesteatoma surgery under endoscopy have a rapid postoperative recovery with significant hearing improvement, and stage IIIA patients can also achieve good results under strict evaluation of indications.

## 1. Introduction

External auditory canal cholesteatoma (EACC) is a cystic mass of skin debris and cholesterol crystals that obstructs the external auditory canal and is not a true tumor with osteoplastic properties. It is an uncommon, benign disease of unclear etiology and pathogenesis. EACC has been reported as a result of external ear canal trauma, chronic inflammation, narrowing of the ear canal, or spontaneous occurrence [1, 2]. Patients with EACC often complain of unilateral ear leakage and otalgia. Unilateral hearing impairment is rarely reported [3, 4]. Patients with EACC initially have limited lesions, mainly present in the external auditory canal, with no obvious symptoms, but when the lesions develop progressively, invading the tympanic membrane into the tympanic chamber and even more into the mastoid process, the facial nerve and extratemporal bone structures are destroyed, and facial nerve palsy and vagal fistulae will inevitably appear. And advanced infiltration of the skull base can cause meningitis or intracranial abscesses [5, 6].

The initial presentation of EACC relies on simple examinations such as frontoscopy and endoscopy, which do not reveal the full extent of the disease [7, 8]. High-resolution temporal bone CT can clearly show the lesion, such as whether it invades the facial nerve or the jugular venous bulb [9, 10]. Shin et al. classified EACC into four types based on the CT of the temporal bone and its clinical features: stage I: lesions limited to the external auditory canal; stage II: lesions invading the tympanic membrane and then protruding into the middle ear; stage III: lesions not limited to the auditory canal and invading the mastoid process; stage IV: lesions not only invading the temporal bone but also involving its adjacent parts [11, 12] (Figure 1).

The principles of treatment for EACC are to completely remove the lesion, maintain normal structure and function, restore the normal epithelial migration ability of the external auditory canal, and maintain the integrity of the tympanic membrane and auditory chain as much as possible. The specific surgical approach should be determined by the extent of the lesion and the specific intraoperative situation. Shin's staging not only evaluates the preoperative site and extent of EACC invasion but also provides a basis for the operator to choose the appropriate surgical approach. Due to the physiological curvature of the external auditory canal or scar stenosis, some relatively hidden lesions (e.g., tympanic cavity and mastoid process) are not clearly identified during microscopic surgery, and there are certain blind spots in the field of view. In contrast, microscopic surgery, in order to remove the hidden lesions present in a wide range of lesions and to preserve important structures, is inevitably achieved at the cost of destroying more bony structures; however, this cost, although we now have many reconstruction methods to repair the relevant structures, is still fraught with difficulties, and the repair does not guarantee the integrity of the original anatomical structures [13, 14].

Based on this, this paper retrospectively analyzed 85 cases of EACC admitted to the Department of Otolaryngology, School of Otolaryngology, Shanghai Jiao Tong University, from January 2016 to February 2021, followed by a retrospective analysis of clinical data to investigate the feasibility and clinical characteristics of total oral endoscopic EACC surgery. A total of 85 EACC patients (90 ears) with a mean age of 49.93 ± 14.87 years were included in the study. According to Udayabhanu staging, 43 ears (47.78%) were stage I, 40 ears (44.44%) were stage II, and 7 ears (7.78%) were stage III. All patients underwent transendoscopic surgery, to explore the different stages of endoscopic otolaryngoscopy surgical approach and efficacy of EACC.

## 2. Materials and Methods

### 2.1. General Clinical Data

General data of cases: a total of 85 (90 ears) EACC cases were included in this study. There were 31 males and 54 females, aged 14-93 years, with age of 50 ± 15 years. The distribution was more concentrated in the two age groups of 14~33 years and 53~71 years. The disease course ranged from 1 week to 30 years, with an average of 31 ± 13 months. Among them, 80 had monaural disease and 5 had binaural disease. 52 ears were left and 38 ears were right. 83 ears (92%) were acquired primary and 7 ears (8%) were secondary. It was secondary to an external auditory canal mass in 2 ears, secondary to external auditory canal atresia in 1 ear, and secondary to radiotherapy for nasopharyngeal carcinoma in 4 ears. The chief complaints were ear stuffiness in 54 patients, earache in 48 patients, hearing loss in 55 patients, tinnitus in 12 patients, ear discharge in 15 patients, ear bleeding in 5 patients, ear itching in 6 patients, and mouth opening pain in 4 patients. None of the patients had vertigo or facial paralysis. 53 patients had experienced one or more external auditory canal irrigations in the outpatient clinic. Otoendoscopy showed granulation in the external auditory canal in 17 cases and a mass in the external auditory canal in 2 cases. All patients underwent middle ear and mastoid CT, and 29 patients (32 ears) underwent pure tone threshold audiometry before surgery. Hearing subjects were normal in 5 ears, conductive deafness in 10 ears, mixed deafness in 12 ears, and sensorineural deafness in 5 ears.

The same skilled otosurgeon performed all the procedures on the study subjects. The hospital medical ethics committee has approved this clinical study, and all patients and their families have given informed consent and signed the informed consent form.

#### 2.1.1. Inclusion Criteria

(1) Medical history is consistent with the clinical presentation of external auditory cholesteatoma. (2) Age is 18-60 years. (3) There is no previous history of otitis media surgery. (4) On examination, visual or endoscopic examination showed white, gray, or brown soft tissue masses and granules in the external auditory canal. (5) On ancillary examination, high-resolution CT of the temporal bone showed soft tissue masses in the external auditory canal with or without destruction of the external auditory canal wall and/or mastoid, destruction of the tympanic chamber, and destruction of the bone wall mainly in the external auditory canal. (6) On audiometry, pure tone audiometry showed conductive deafness or mixed deafness. (7) Pathological diagnosis is external auditory canal cholesteatoma.

#### 2.1.2. Exclusion Criteria

Exclusion criteria are as follows: (1) significant narrowing and malformation of the external auditory canal; (2) benign and malignant tumors and tuberculosis of the external auditory canal; (3) mental disorders, cognitive and consciousness disorders; (4) serious underlying diseases with poor control (e.g., diabetes, coagulation disorders, and malignant tumors); (5) pregnant or preparing for pregnancy, lactating; and (6) unable to cooperate with the evaluation.

### 2.2. Research Methods

All patients underwent otoendoscopy, CT of the middle ear and mastoid, and otoendoscopic surgical treatment. According to the extent of lesion invasion in EACC, Udayabhanu staging was adopted [15]. Stage I: the lesion is confined to the external auditory canal without bone destruction; stage II: there is bone destruction with or without middle ear involvement, but does not involve adjacent structures (including temporomandibular joint, mastoid process, jugular bulb, facial nerve bone canal, and dura mater); stage IIIA: those with bone destruction and involvement of adjacent structures, but no complications; stage IIIB: those with other complications at the same time. In this study, 43 ears were in stage I, 40 ears were in stage II, and 7 ears were in stage IIIA according to the Udayabhanu stage. There were 31 ears with otitis externa, 4 ears with secretory otitis media, 10 ears with tympanic membrane perforation, and 1 ear with external auditory canal atresia; see Table 1.

### 2.3. Treatments

All patients underwent ESS under local or general anesthesia. Among them, 64 patients (67 ears) underwent local anesthesia surgery (39 ears in stage I, 24 ears in stage II, and 4 ears in stage IIIA) and 21 patients (23 ears) underwent general anesthesia surgery (4 ears in stage I, 16 ears in stage II, and 3 ears in stage IIIA). Intraoperative diagnosis combined with CT and intraoperative findings showed destruction of the bone wall of the external auditory canal in 47 ears (40 ears in stage II and 7 ears in stage IIIA). Among them, 31 had destruction of the posterior wall of the ear, 28 had destruction of the inferior wall of the ear, 26 had destruction of the anterior wall of the ear, and 19 had destruction of the parietal wall of the ear. There were 19 ears with annular destruction of the bone wall of the external auditory canal, 29 ears with thin invagination of the tympanic membrane, 10 ears with perforation of the tympanic membrane, and 4 ears with destruction of the ossicular chain. It involved the horizontal and vertical segments of the facial nerve canal in 1 ear, the temporomandibular joint in 5 ears, and the mastoid process in 1 ear. 74 ears underwent exclusively otoendoscopic resection of EACC, 2 ears underwent otoendoscopic resection of EACC+resection of external auditory canal mass, 3 ears underwent otoendoscopic resection of EACC+tympanoplasty, 9 ears underwent otoendoscopic resection of EACC+tympanoplasty+tympanoplasty, 1 ear underwent otoendoscopic resection of EACC+tympanoplasty, and 2 ears underwent otoendoscopic resection of EACC+atticotomy+tympanoplasty+ossicular chain reconstruction (PORP 1 ear, autologous ossicles 1 ear).

Among them, 7 ears were repaired with tragus cartilage-perichondrium and 2 ears were repaired with tragus perichondrium.

### 2.4. Procedures

1. Local anesthesia and preoperative preparation: patients with local block anesthesia of the external auditory canal combined with external auditory canal mass underwent tumor resection
2. Exploration and resection of cholesteatoma: for impacted significant cholesteatoma, the volume was first reduced from the center of the lesion and then the dissection was performed between the cholesteatoma capsule and the external auditory canal skin until the pocket was completely removed
3. Thorough cleaning of the epithelium: sequential cleaning of the epithelium at the “pit” of bone destruction, the epithelium around the tympanic ring, and the epithelium and granulation on the surface of the tympanic membrane. The tympanic membrane was checked for integrity. There was pinpoint perforation or small perforation of the tympanic membrane with exudation, and preoperative CT showed no significant abnormality of the tympanum, which was not repaired at the same time. Tympanic exploration was performed while moderate or large perforation of the tympanic membrane or preoperative CT revealed tympanic soft tissue shadows
4. Exploration of the tympanum: an external auditory canal skin tympanic membrane flap was done and the exploration tympanum was lifted. If there was cholesteatoma epithelium in the tympanic cavity, incision and exploration of the lateral wall of the attic were performed. If the ossicular chain is interrupted/destroyed, the corresponding reconstruction is performed. For patients with attic incision, the tragus cartilage-perichondrium was used to repair the residual tympanic membrane, while for patients with tympanic membrane perforation, the tragus perichondrium was used to repair the residual tympanic membrane
5. Reconstruction of the ossicular chain: there was ossicular chain destruction for corresponding artificial ossicular chain reconstruction

## 3. Results

All patients in this study had no statistical differences in general data indicators such as age of onset, side, and gender and were balanced and comparable, and the clinical characteristics are shown in Table 1. All patients were pathologically confirmed to have EACC after surgery. Referring to the typology of foreign scholars Naim [3, 8] and domestic scholars Huang Hongming [16], a total of 85 patients with EACC (90 ears) were included in this study, with a mean age 49.93 ± 14.87 years. According to Udayabhanu staging, 43 ears (47.78%) were stage I, 40 ears (44.44%) were stage II, and 7 ears (7.78%) were stage III. All patients were discharged the day after surgery and were reviewed regularly at 1 week, 2 weeks, 1 month, 3 months, and 6 months postoperatively. All patients were followed up regularly for 12 to 68 months. One patient with EACC stage II and external auditory atresia recurred 6 months after surgery and underwent endoscopic tympanoplasty+tympanoplasty+auditory chain reconstruction again. Eight months after the second surgery, the localized lesion in the external auditory canal recurred again and an endoscopic removal of EACC was performed, which has been recurrence-free for 12 months. One patient with stage II disease recurred 12 months after surgery and again underwent endoscopic resection of the EACC and has been recurrence-free for 9 months. The rest of the patients have been followed up with no recurrence.

## 4. Discussion

### 4.1. Endoscopic Options for Different Stages of EACC

Udayabhanu proposed the following staging criteria for EACC: stage I lesions are limited to the external auditory canal without bone destruction, stage II lesions are those with bone destruction with or without middle ear involvement but without the involvement of adjacent structures (including the temporomandibular joint, mastoid process, jugular venous bulb, facial nerve canal, and dura mater), stage IIIA lesions are those with bone destruction and involvement of adjacent structures without complications, and stage IIIB lesions are those with a combination of other complications [17]. Unlike the classical Holt staging, which includes the area of invasion of the middle and upper tympanic chambers, which are the areas of predominance for endoscopic surgery, stage III of Holt staging is relatively broad. Compared with Holt's staging criteria, stage II patients have a larger scope (e.g., superior tympanic chamber), and for the current endoscopic management of superior tympanic cholesteatoma [18], stage II patients of Udayabhanu can be completely resolved, and some stage IIIA patients are also feasible for endoscopic surgery after comprehensive evaluation, but strict indications need to be mastered, and timely replacement of the posterior auricular approach with microscopic mastoid surgery should be prepared. There is preparation of the posterior auricular access microscopic mastoid surgery. In the three stage IIIA patients in this study, one case did not invade the temporomandibular joint, so the operation was performed in the same way as in stage II patient; two patients with invasion of the mastoid cavity required mastoid opening, and endoscopic mastoid opening was chosen because the mastoid in these two cases was of the plate-barrier type, and the mastoid air space only had a small cavity, so it was not necessary to remove a large amount of bone in a small space, and the patient was prepared to change the microscope at any time. In patients with good mastoid pneumatization and lesions involving most of the mastoid airspace or even the mastoid tip, endoscopic opening of the mastoid is not recommended. In the current literature, it is recommended to perform external auditory canal formation after removal of cholesteatoma in adults with EACC [19], because the external auditory canal of patients with EACC is mostly in the shape of a “flask” with a large inner and small outer surface after removal of cholesteatoma, which may cause postoperative narrowing and recurrence of the external auditory canal. In the present study, there was no recurrence in any of the cases, and only one case of membranous atresia, which was recanalized after repeated cautery with silver nitrate.

### 4.2. Case Characteristics

The clinical incidence of EACC is low, and the first diagnosis in the outpatient clinic is less confirmed. In this study, 53 patients (62%) experienced at least one outpatient irrigation treatment with impacted cerumen as the first diagnosis, which may be related to cerumen accumulation on the keratinocyte surface in some patients with cholesteatoma. The maximum number of rinses was 5, which may be related to insufficient experience in diagnosis and treatment in lower community hospitals. Given the different incidence ratio between men and women, reports vary in the literature. There were 31 males (36%) and 54 females (64%) in this study. Both the age of onset and the course of the disease present a polarization. There were more adolescent patients and elderly patients and more patients with disease duration of less than 1 month and more than 10 years. It may be due to the narrower external auditory canal in younger patients and decreased epithelial migration and poor hygiene in older patients. 45 (53%) patients had an onset time of no more than 1 month and were mostly accompanied by ear stuffy ear pain, which was associated with acute infection or periostitis of the external auditory canal caused after irrigation stimulation. Nine (11%) patients had an onset time of more than 10 years, which was considered to be related to the fact that the patients did not return after anti-infective treatment in the acute phase and their willingness to seek treatment decreased. Acquired primary in 83 ears (92%), secondary in 7 ears (8%), secondary to external auditory canal mass in 2 ears, secondary to external auditory canal atresia in 1 ear, and secondary to nasopharyngeal carcinoma after radiotherapy in 4 ears. The relationship between a history of radiotherapy for NPC and the incidence of EACC has rarely been mentioned in previous literature. In fact, we found that EACC patients with a history of radiotherapy for nasopharyngeal carcinoma were mostly associated with secretory otitis media, which was associated with radiation damage to the cilia of the middle ear mucosal epithelium and decreased self-cleaning ability of the external auditory canal skin; see Figure 2.

### 4.3. Extent of Disease and Direction of Invasion

CT of EACC showed soft tissue shadows in the external auditory canal with/without bone destruction, with/without middle ear involvement. It has been reported in the literature that its growth direction shows an “inward roll” property characterized by outside-in, which is distinguished from inside-out of middle ear cholesteatoma. EACC may involve the attic and tympanic sinuses inward or the mastoid posteriorly. In this study, the posterior wall was the most destroyed in statistics, which is more consistent with literature reports.

There are two main directions of external auditory canal cholesteatoma invasion. The tympanic membrane is compressed inward, resulting in thin, invaginated, loss of elasticity, and even perforation of the tympanic membrane. If some patients have repeated irrigation or coinfection, it can also cause acute inflammation or even perforation of the tympanic membrane. In this study, 10 ears (12%) had perforation. The cholesteatoma epithelium enters the attic and tympanic sinuses through perforation and destroys structures such as the ossicular chain, which can involve the horizontal segment of the facial nerve canal. The other is the mastoid posteriorly, involving the vertical segment of facial nerve canal; see Figure 3.

For middle ear cholesteatoma, the facial nerve is most commonly involved in the horizontal and conical segments. For EACC, the most commonly affected facial nerve is the vertical segment, as it can invade the mastoid process. Four ears had secretory otitis media in this study. After EACC destroys the external auditory canal, the wall will block the mastoid air cells, poor drainage causes mastoid effusion, and nasopharyngeal carcinoma radiotherapy complicated by secretory otitis media is much common. Endoscopic surgery does not involve bone grinding in the mastoid region and cannot expose the entire course of the facial nerve canal, so endoscopic surgery should pay attention to avoid injury in patients with EACC involving the mastoid process, especially those with bone destruction in the mastoid segment of the facial nerve canal suggested by preoperative CT.

### 4.4. Selection of Surgical Plan and Skills

#### 4.4.1. Selection of Anesthesia

64 patients (67 ears: 39 ears in stage I, 24 ears in stage II, and 4 ears in stage IIIA) were operated on with local anesthesia. 21 patients (23 ears: 4 ears in stage I, 16 ears in stage II, and 3 ears in stage IIIA) were operated on with general anesthesia. In this study, we found that stage I and II can be completely operated with local anesthesia, while some stage II and IIIA patients involving attic chiseling were recommended for general anesthesia surgery. For patients with external auditory canal cholesteatoma, the effect of local block anesthesia of the external auditory canal was inferior to that of tympanic membrane repair under local anesthesia because they have experienced repeated ear canal irrigation, combined otitis externa, and external auditory canal periostitis in the outpatient clinic. Most of the patients with tympanic membrane repair under local anesthesia had no pain. In external auditory canal cholesteatoma surgery under local anesthesia, about 20% of patients complain of pain during surgery, which was mostly tolerable. Only one 91-year-old female patient complained of intolerable ear pain. For such patients, in addition to local block anesthesia of the external auditory canal, local block anesthesia of the posterior auricular sulcus and temporomandibular joint fossa can be added, and attention should be paid to the direction and depth of needle insertion to implement injection to avoid causing transient facial paralysis [20]. During the operation, the patient's mood can be soothed by communicating with the patient, encouraging positively, and playing music. In this study, 4 juvenile patients (3 under general anesthesia and 1 under local anesthesia) were enrolled. General anesthesia is recommended for minor patients to avoid emotional stress, pain, and inability to cooperate to complete the operation or psychological shadow. For stage IIIA and IIIB patients, general anesthesia is recommended for surgery, due to the possibility of conversion to microscopic open surgery during surgery.

#### 4.4.2. Surgical Options

In stage I patients with EACC, otoendoscopic resection of external auditory canal cholesteatoma was performed, and those with external auditory canal tumors also underwent resection of external auditory canal tumors. Patients with EACC stage II and secretory otitis media underwent otoendoscopic resection of external auditory canal cholesteatoma+tympanic membrane. There are not many reports on this in the previous literature, considering that the patients with personal history of nasopharyngeal carcinoma in this study were caused by decreased epithelial self-cleaning ability due to radiotherapy. For patients with EACC stage II~III, otoendoscopic resection of external auditory canal cholesteatoma+tympanic exploration+tympanoplasty (+ossicular chain reconstruction) was performed.

In EACC stage III, even if mastoid was involved, most were cholesteatoma invasion and obstructive inflammation. Mastoid inflammation can improve spontaneously after thorough epithelial cleaning and unobstructed drainage. Not many cases of this have been reported. There are a large number of domestic reports on EACC [21], especially stage III. However, the number of reported cases of stage III ESS is less [22].

#### 4.4.3. Recurrence

There were a total of 2 patients with recurrence in this study.

One of the patients with recurrence had atresia of the external auditory canal, and the first operation was performed under otoendoscope to chisel the atretic bone, clean the external auditory canal and tympanic cholesteatoma epithelium, and perform tympanoplasty. The patient's own ear canal was narrow and recurred again after surgery; thus, epithelial debridement under local anesthesia was performed. The principle of surgical treatment of EACC is complete removal of the lesion, followed by reconstruction of the external auditory canal structure to restore epithelial self-cleaning ability. Patients with recurrent cholesteatoma in the literature are mostly associated with external auditory canal stenosis or atresia, and microscopic external auditory meatoplasty is recommended. If some narrow lesions of the external auditory canal are present for more than 1/2 week, external auditory canal skin grafting is considered [23]. Therefore, ESS has limitations for the treatment of patients with external auditory canal stenosis.

### 4.5. Advantages of Endoscopic EACC Surgery

For stage I and II EACC patients with invasion of the external auditory canal bone and tympanic membrane, endoscopic surgery is the best choice, and with the increasing use of endoscopy in middle ear surgery, it has the advantages of aesthetics, faster postoperative recovery, smaller visual field blindness, and more direct surgical access compared to traditional microsurgery with posterior or internal ear incisions [24]. In the present study, six patients with invasion of the tympanic cavity had no significant exudation after removal of the ear canal filling 14 days after surgery, and the tympanic membrane and external auditory canal skin grew well 1 month after surgery. For patients with stage IIIA invasion of the mastoid, it takes about 3 months for the dry ear to open after microscopic mastoid root treatment with posterior ear access, and there is no improvement or decrease in hearing [25]. In this study, there was no significant exudation after removal of the ear canal filling at 14 days in stage IIIA patients, and the tympanic membrane and external ear canal skin grew well at 1 month after surgery, and the average postoperative air-conduction hearing improved and the air-bone conduction difference decreased significantly.

In conclusion, patients with stage I and II external auditory canal cholesteatoma recovered quickly after endoscopic surgery and had significantly improved hearing, and the air-bone conduction difference was significantly reduced or disappeared, while stage IIIA patients could also achieve good results under strict evaluation of indications, but should be prepared to change microscopic surgery at any time. However, the sample size of this study was small, a more comprehensive understanding of the use of endoscopy in patients with stage III external auditory canal cholesteatoma is lacking, and a larger sample is needed to evaluate the effectiveness of staged treatment.

## 5. Conclusion

Although it is a nongenuine tumor, it is biologically aggressive, easily destroying bone and eroding adjacent structures. The preoperative imaging (temporal bone resolution CT) is an important clinical guide for otologists to assess the extent of lesion destruction, diagnose EACC, guide clinical staging, and select the appropriate surgical approach. Patients with stage I and II EACC can be completely managed endoscopically, and most patients can even tolerate local anesthesia, and patients with disrupted auditory chain can undergo simultaneous or two-stage reconstruction. Some stage IIIA EACC patients can be operated endoscopically and require simultaneous tympanoplasty+tympanoplasty (+auditory chain reconstruction). Some stage IIIA and IIIB cases require microscopic management or combined surgery with laparoscopy. ESS has limitations in cases with external auditory canal stenosis, and microscopic external auditory meatoplasty is recommended.

## Figures and Tables

**Figure 1:** CT images of the Shin stages of EACC. Note: (a) stage I: soft tissue shadow in the right external auditory canal, the lesion is confined to the external auditory canal without bone destruction; (b) stage II: soft tissue shadow in the left external auditory canal invades the tympanic membrane into the middle ear cavity and destroys the bone of the external auditory canal wall; (c) stage III: soft tissue shadow in the right external auditory canal, not only destroys the bone of the external auditory canal but further invades the small bone of the middle ear cavity and involves the mastoid.

**Figure 2:** Excision of external auditory canal cholesteatoma in patients with EACC stage II. Note: (a) CT in patients with EACC stage II revealed destruction of the bone wall of the external auditory canal and no involvement of the middle ear; (b) cerumen and white cholesteatoma epithelium in the external auditory canal were observed under an otoendoscope; (c) ear endoscopy after external auditory canal cholesteatoma removal surgery in patients shows intact and thin tympanic membrane and enlargement of the bone wall of the external auditory canal.

**Figure 3:** CT of EACC stage III patients (white arrow: the vertical segment of the facial nerve is destroyed and exposed).

**Table 1:** Clinical data and result analysis of 85 cases (90 ears) of EACC.

—	—	Number of samples	Percentage
Patients	Cases	85	—
—	Ears	90	—
Sex	—	—	—
—	Male	31	36%
—	Female	54	64%
Age	—	—	—
—	Minimum	14	—
—	Maximum	93	—
Sides	—	—	—
—	Left	52 (ears)	58%
—	Right	38 (ears)	42%
Monaural	—	—	—
Binaural	Monaural	80 (ears)	94%
—	Binaural	5 (ears)	6%
Acquired primary/secondary	—	—	—
—	Primary	83 (ears)	92%
—	Secondary	7 (ears)	8%
Secondary disease	—	—	—
—	External auditory canal tumor	2 (ears)	2%
—	Atresia of external auditory canal	1 (ear)	1%
—	After radiotherapy for nasopharyngeal carcinoma	4 (ears)	4%
Clinical features	—	—	—
—	Ear stuffiness	54	64%
—	Ear pain	48	567%
—	Hearing loss	55	65%
—	Tinnitus	12	14%
—	Ear discharge	15	18%
—	Ear bleeding	5	6%
—	Ear itching	6	7%
—	Ear mouth opening pain	4	5%
Hearing condition	—	—	—
—	Normal	5 (ears)	6%
—	Conductive deafness	10 (ears)	11%
—	Mixed deafness	12 (ears)	13%
—	Sensorineural hearing loss	5 (ears)	6%
Udayabhanu stage			
—	I	43 (ears)	48%
—	II	40 (ears)	44%
—	IIIA	7 (ears)	8%
—	IIIB	0	0
Combined with other diseases of middle ear and external ear	—	—	—
—	Otitis externa	31 (ears)	34%
—	Secretory otitis media	4 (ears)	4%
—	Tympanic membrane perforation	10 (ears)	11%
—	Atresia of external auditory canal	1 (ear)	1%
Anesthesia	—	—	—
—	Local	64 (67 ears)	75% (74%)
—	General	21 (23 ears)	25% (26%)
Ossicular chain reconstruction	—	—	—
—	No	88 (ears)	98%
—	PORP	1 (ear)	1%
—	TOPR	0 (ear)	0
—	Autogenous ossicles	1 (ear)	1%

## Data Availability

The figures and tables used to support the findings of this study are included in the article.
